The article "The Efficacy of Health Surveys and Polymerase Chain Reaction Tests Prior to Judo Tournaments During the COVID-19 Pandemic" was published in 2022. Journal: Cureus.

# The Efficacy of Health Surveys and Polymerase Chain Reaction Tests Prior to Judo Tournaments During the COVID-19 Pandemic

**DOI:** 10.7759/cureus.20882

**Published:** 2022-01-02

**Authors:** Naoki Sakuyama, Yasuo Mikami, Akira Ikumi, Naohisa Fujita, Shinji Nagahiro

**Affiliations:** 1 Medical Science Committee, All Japan Judo Federation, Bunkyo, JPN; 2 Surgery, Tobu Chiiki Hospital, Tokyo Metropolitan Health and Medical Treatment Corporation, Katsushika, JPN; 3 Rehabilitation Medicine, University Hospital, Kyoto Prefectural University of Medicine, Kyoto, JPN; 4 Orthopedic Surgery and Sports Medicine, Tsukuba University Hospital Mito Clinical Education and Training Center, Mito, JPN; 5 Infection Control and Laboratory Medicine, Kyoto Prefectural Institute of Hygienic and Environmental Sciences, Kyoto, JPN; 6 Neurosurgery, Yoshinogawa Hospital, Tokushima, JPN

**Keywords:** covid-19, tournament, health survey, pcr test, judo

## Abstract

Background

As of October 2021, sports activities require preventive measures against coronavirus disease 2019 (COVID-19) infection. Judo, a close-contact sport, demands careful prevention with great consideration to the risk of infection. The All Japan Judo Federation Medical Science Committee (AJJF) designed COVID-19 prevention protocols from a medical perspective and developed policies for safe regular practices and tournaments.

Objective and Methods

We aim to examine the efficacy of health surveys and polymerase chain reaction (PCR) tests prior to judo tournaments, as mandated by the tournament policy. Infection prevention managers were installed prior to tournaments. Two weeks prior to each tournament, these managers drafted health inventory forms for athletes and related parties to check for COVID-19-associated symptoms. Although PCR testing prior to tournaments was not required by policy, the AJJF conducted them (directly and by mail) prior to six tournaments from October 2020 to September 2021 for athletes whose health inventory forms listed no symptoms.

Results

One of the athletes was not tested and was unable to participate in a tournament due to the symptoms indicated in their health inventory form. Testing began in October 2020 and was conducted until September 2021 for 2,073 athletes over the duration of six tournaments. The SARS-CoV-2 virus was detected in 11 (0.29%) athletes. In tournaments held until April 2021, SARS-CoV-2 was detected in only one of the 1,173 (0.08%) athletes tested. However, prior to tournaments held from July 2021 onward, when variants became prevalent, SARS-CoV-2 was detected in 10 (1.1%) of the 900 athletes tested (p < 0.05). No clusters were reported in association with any tournament.

The article "The Efficacy of Health Surveys and Polymerase Chain Reaction Tests Prior to Judo Tournaments During the COVID-19 Pandemic" was published in 2022. Journal: Cureus.

Conclusion

We believe that drafting health inventory forms two weeks prior to judo tournaments was essential and kept the participants alert. However, as variants emerged, some participants who were positive could not be detected through their inventory forms; this demonstrates the need for caution when relying on health inventory forms alone.

## Introduction

The first coronavirus disease 2019 (COVID-19) infections were reported in China in January 2019 [1] and subsequently expanded into a pandemic [2]. In Japan, a string of regions was forced to declare states of emergency due to high infection rates [3]. Furthermore, the COVID-19 pandemic has greatly affected sports. Globally, many sporting bodies such as the National Collegiate Athletic Association in the United States have drafted guidelines for preventing COVID-19 infections [4,5]. COVID-19 responses for contact sports such as rugby and American football have allowed those sports to gradually resume play [6]. Judo is also a contact sport, but it involves an especially high level of close contact. To address this, the International Judo Federation has issued required protocols during the COVID-19 pandemic [7].

Having considered protocols for preventing infections in the close-contact sport of judo, we at the All Japan Judo Federation Medical Science Committee (AJJF) drafted guidelines for holding judo competitions and presented them to dojos and instructors throughout Japan [8]. In addition to enforcing these protocols for judo practice, we also felt it necessary to implement them for tournaments. When holding tournaments in which athletes gather from all areas of Japan, we settled on a policy to inhibit the spread of COVID-19 using health survey forms prior to tournaments to screen for athletes at risk of COVID-19 infection and to prohibit them from participating, followed by polymerase chain reaction (PCR) tests for all remaining athletes.

To our knowledge, no previous study has examined COVID-19 infection in tournaments where the above measures were implemented. We thought of examining health surveys and PCR tests prior to tournaments and that we could hold the tournaments without the infected athletes. In this study, we aim to verify the efficacy of conducting health surveys and PCR tests prior to judo tournaments in preventing COVID-19 infection.

## Materials and methods

The present study was conducted with approval from the Institutional Review Board of Tobu Chiiki Hospital. Upon the decision to hold a tournament, we asked all participating athletes and other associated parties to complete a health inventory form every day beginning two weeks prior to the date of the tournament. When we conducted this study, all athletes did not inoculate the vaccine of COVID-19.

The article "The Efficacy of Health Surveys and Polymerase Chain Reaction Tests Prior to Judo Tournaments During the COVID-19 Pandemic" was published in 2022. Journal: Cureus.

The health inventory forms asked questions related to the primary symptoms of COVID-19. Data collected included body temperature, coughing, sneezing, sore throat, taste dysfunction, distorted sense of smell, malaise, diarrhea, vomiting, abdominal pain, and respiratory distress [9]. For body temperature, individuals completing the forms calculated their average body temperature over two weeks. A body temperature <0.5°C higher than the average was considered normal body temperature, while a body temperature ≥0.5°C higher than the average was considered a fever.

Athletes were asked to refrain from training outside their own dojos for two weeks prior to a tournament. PCR tests were conducted one to seven days prior to tournaments with either real-time PCR (RT-PCR) or loop-mediated isothermal amplification (LAMP) with saliva. On the day of the PCR test, the athlete’s health inventory form was checked. If any abnormalities were found, the PCR test is not conducted, and the athlete was deemed ineligible to enter the tournament and asked to undergo examination at a hospital.

Participants were also considered ineligible for PCR tests if their health inventory forms indicated at least three consecutive days of symptoms at any point up to one week prior to testing, at least two consecutive days of symptoms one week to four days prior to testing, or at least one day of symptoms within the past three days. These stipulations were also applied upon entry to the tournament venue. Anyone with symptoms, even if their PCR test result was negative, was barred from entering the tournament venue.

In cases in which teams have athletes who were infected within two weeks prior to a tournament, individuals who tested positive were not allowed to participate. Athletes in close contact with the infected person within two weeks prior to a tournament were barred from participating. The remaining athletes on the same team were allowed to participate if their PCR test results were negative.

In accordance with the guidelines set by the Japanese Ministry of Health, Labour and Welfare, a person in close contact was defined as follows: 1) a person living with or having a long period of contact (including being in the same car, aircraft, etc.) with a patient (confirmed case); 2) a person with a high likelihood of having had direct contact with respiratory secretions, bodily fluids, or other contaminants of a patient (confirmed case); or 3) a person in contact with a patient (confirmed case) within touching distance (roughly 1 m) for at least 15 minutes (transmissibility is assessed comprehensively based on factors such as the surrounding environment and the nature of contact).

The article "The Efficacy of Health Surveys and Polymerase Chain Reaction Tests Prior to Judo Tournaments During the COVID-19 Pandemic" was published in 2022. Journal: Cureus.

In the event of a positive PCR test prior to a tournament, the athlete was immediately sent to a hospital for diagnosis and registered at a public health center for management. Athletes were tested again at a medical center if there were suspected false positive or inconclusive results. If the result was negative, they were allowed to participate in the tournament. Infection records were followed up in the cohort for two weeks after a tournament. Anyone who developed COVID-19 in association with a tournament was registered at a public health center (Figure 1).

**Figure 1:** Flowchart of the study

We divided athletes into two groups: the Non-Mutant Group (NMG), who underwent tests from the start of testing in Japan until June 2021, and the Mutant Group (MG), who underwent tests from July 2021 onward, when variants of SARS-CoV-2 became prevalent.

Statistical analysis

The associations between the NMG and MG were evaluated using Pearson’s χ2 test. All calculated p-values were two-sided, and statistical significance was set at p < 0.05. All statistical analyses were performed using the JMP 13 software (SAS Institute, Cary, NC, USA).

## Results

A total of 2,073 athletes were tested prior to six individual tournaments held between October 2020 and September 2021. Prior to the first two of these tournaments, PCR tests were conducted on-site for the four subsequent tournaments, and testing was conducted by mail.

Testing was performed with RT-PCR for 1,140 athletes (55%) and with LAMP for 933 athletes (45%). The 2,073 athletes consisted of 1,106 men and 967 women, with a median age of 18 years (16−35 years) (Table 1).

**Table 1:** Athletes’ background *Median (range)

n	2,073
Number of tournaments	6
Testing pattern in the tournaments (direct testing/by mail)	2 (33.3%)/4 (67.7%)
Real-time PCR (RT-PCR)	1,140 (55%)
Loop-mediated isothermal amplification (LAMP)	933 (45%)
Male/female	1,106 (53.4%)/967 (46.6%)
Age*	18 (16–35)

One athlete was deemed ineligible for a PCR test on the day of testing based on their health inventory form.

A total of 22 athletes (1.06%) were unable to undergo PCT testing due to having developed COVID-19, having been confirmed to be in close contact with an infected person, or having a teammate who was infected or was in close contact with an infected person. A total of 46 athletes (2.2%) were unable to participate in tournaments due to COVID-19-related withdrawals prior to the tournaments. PCR tests detected the SARS-CoV-2 virus in 11 athletes (0.53%). Two athletes (0.096%) developed COVID-19 within 48 hours after a tournament. Another 11 athletes (0.53%) developed COVID-19 48 hours to 14 days after a tournament (Figure 2).

The article "The Efficacy of Health Surveys and Polymerase Chain Reaction Tests Prior to Judo Tournaments During the COVID-19 Pandemic" was published in 2022. Journal: Cureus.

**Figure 2:** Flowchart of the PCR test results

We compared two groups of athletes as follows: the NMG (n = 1,173), who underwent tests from the start of testing in Japan until June 2021, and the MG (n = 900), who underwent tests from July 2021 onward, when variants of SARS-CoV-2 were prevalent.

PCR tests detected SARS-CoV-2 more frequently in the MG (n = 10; 1.1%) than in the NMG (n = 1; 0.08%). This difference was significant (p < 0.05). PCR testing was deemed inapplicable based on health inventory forms for one athlete in the NMG (0.08%) versus no athletes in the MG. This difference was not significant. PCR testing was deemed inapplicable due to reasons such as prior infection or close contact for five athletes in the NMG (0.43%) versus 16 athletes in the MG (1.78%); thus, this ineligibility was significantly more common in the MG (p < 0.05). COVID-19 developed within 48 hours after a tournament in no athletes in the NMG versus two athletes in the MG (0.1%). This difference was not significant. However, 3−14 days after a tournament, COVID-19 developed significantly more frequently in the MG (n = 9; 1%) than in the NMG (n = 2; 0.17%) (p < 0.05) (Table 2).

**Table 2:** Results of comparison between Non-Mutant Group and Mutant Group *p < 0.05.

n = 2,073	Non-Mutant Group (NMG) (October 2020–June 2021)	Mutant Group (MG) (July 2021–September 2021)	p
Number of tests	1,173	900	0.58
Positive tests	1 (0.08%)	10 (1.1%)	0.0007*
Ineligible cases for health inventory forms	1 (0.08%)	0	0.38
Tournament participation refusal for the prior infection	5 (0.43%)	16 (1.78%)	0.0023*
Post-tournament infections within 48 hours	0	2 (0.1%)	0.37
Post-tournament infections 48 hours to 14 days	2 (0.17%)	9 (1%)	0.0026*
Highest infection index in Japan/100,000 people (month/year)	122.68 (1/2021)	443.14 (8/2021)	<0.0001*

No clusters were reported in association with any tournaments.

## Discussion

As of November 2021, the total number of reported COVID-19 infections worldwide was roughly 247 million, with roughly five million deaths [2,10]. Amidst the COVID-19 pandemic, athletic organizations in various sports have rapidly drafted guidelines for preventing and managing infections [5,11]. The National Collegiate Athletic Association and rugby were quick to draft guidelines and have been on the forefront of contact sports regarding new protocols [4,12,13].

In judo, which involves throws and ground grappling, close contact is unavoidable. Consequently, judo requires stricter infection prevention measures than other sports. In April 2020, we issued COVID-19 infection prevention guidelines for judo from a medical science perspective. We have published four revisions of the guidelines since the initial implementation, which have been used to announce protocols for tournaments [8]. The need for PCR tests was left to the discretion of tournament directors, who did not always consider them necessary [14,15]. Tournaments held by the AJJF gather athletes from all over Japan. Determining infection status around the country is difficult, and tournaments require individual athletes’ infection statuses, which prompted us to perform PCR testing. Tests were conducted with saliva tests, which have already been demonstrated to be effective and can be performed more safely than nasopharyngeal swabs [16].

The article "The Efficacy of Health Surveys and Polymerase Chain Reaction Tests Prior to Judo Tournaments During the COVID-19 Pandemic" was published in 2022. Journal: Cureus.

In tournaments held until April 2021, when the highest infection index in Japan was 122.68/100,000 people (January 2021) [17,18], only one out of 1,173 athletes who had undergone PCR testing had tested positive. We believed that prohibiting participation by athletes whose health inventory forms indicated symptoms, athletes who had previously developed COVID-19, and athletes in close contact with infected people would enable tournaments to be held safely. However, in July 2021, while the infection ratios of the wild-type R. 1 variant and α variant of SARS-CoV-2 began to decrease, the infection ratio of the δ variant began to increase [19]. In August 2021, the infection index/100,000 people increased to 443.14, thus surpassing 400 [17,18]. Japan declared the highest emergency alert level. In a tournament held during that period, SARS-CoV-2 was detected in 10 of 900 athletes tested, a figure significantly higher than at any previous tournament.

In addition, a significantly high number of athletes could not undergo PCR tests due to previous infection or being in close contact with infected people (p < 0.05), suggesting that asymptomatic infected people cannot be detected with health inventory forms alone. In the future, it may be necessary to conduct tests selectively on athletes from regions with high infection rates to determine their infection status as a basis for assessing whether all athletes should be tested.

Health surveys and PCR testing, which we examined, could exclude athletes with suspected infection prior to tournaments. No clusters were reported in association with any tournaments. We think that our infection control strategy reduced the risk of infection.

This study has some limitations. Testing was limited to athletes and was not performed on other parties involved in the tournaments. Considering the rate of infection spread, it is necessary to expand testing to involve tournament-related personnel as well. Moreover, at the time of this study, no athlete had been inoculated with the COVID-19 vaccine. When inoculation of the COVID-19 vaccine spread in Japan, it may be necessary to investigate the need for the health surveys and PCR tests of the athletes again.

The article "The Efficacy of Health Surveys and Polymerase Chain Reaction Tests Prior to Judo Tournaments During the COVID-19 Pandemic" was published in 2022. Journal: Cureus.

## Conclusions

We have been able to hold judo tournaments safely during the COVID-19 pandemic by surveying athletes’ health two weeks prior to tournaments. Screening tests may need to be considered in tournament protocol while SARS-CoV-2 variants remain prevalent.
